The article "The NAO Variability Prediction and Forecasting with Multiple Time Scales Driven by ENSO Using Machine Learning Approaches" was published in 2022. Journal: Comput Intell Neurosci.

# The NAO Variability Prediction and Forecasting with Multiple Time Scales Driven by ENSO Using Machine Learning Approaches

**DOI:** 10.1155/2022/6141966

**Published:** 2022-04-15

**Authors:** Bin Mu, Jing Li, Shijin Yuan, Xiaodan Luo

**Affiliations:** Department of Software Engineering, Tongji University, Shanghai, China

## Abstract

Machine learning methods have now become an optional technique in Earth science research, and such data-driven solutions have also made tremendous progress in weather forecasting and climate prediction in recent years. Since climate data are typically time series, the neural network layers, which can identify the intrinsic connections between the points of the sequence and features in two-dimensional data, perform particularly well for climate prediction. The North Atlantic Oscillation (NAO) is a prominent atmospherical mode in the northern hemisphere, with the frequency change characteristic of sea level pressure (SLP) in the North Atlantic sector. One of the reasons why NAO prediction is still challenging is that NAO is also proven to be influenced by other climate circulations, the most significant of which is the interaction between El Niño-Southern Oscillation (ENSO) and NAO. Therefore, sea surface temperature (SST) in the Pacific Ocean used to characterize ENSO is also one of the factors that contribute to the evolution of NAO and can be used as an input factor to predict the NAO. In this paper, the seasonal lag correlation between ENSO and NAO is explored and analyzed. The interaction has been considered in both short-term forecasting and midterm prediction of the NAO variability. The monthly NAO index (NAOI) fluctuation is predicted using the Niño indices based on the RF-Var model, and the accuracy achieves 68% when the lead time is about three months. In addition, integrating multiple physical variables directly related to the NAO and Pacific SST, the short-term NAO forecasting is conducted using a multi-channel neural network named AccNet with trajectory gated recursive unit (TrajGRU) layer. AccNet has the ability to identify the mechanism of the high-frequency variation in several days, and the NAO variability is indicated by SLP. The loss function of AccNet is set to anomaly correlation coefficient (ACC), which is the indicator that verifies spatial correlation in geoscience. Forecasting extreme events of NAO between 2010 and 2021, AccNet presents higher flexibility compared against other structures that can capture spatial-temporal features.

## 1. Introduction

The North Atlantic Oscillation (NAO) is the most prominent phenomenon of atmospheric circulation resulting in sea level pressure (SLP) fluctuation on Azores and Iceland [1]. The weather and climate in the Euro-Atlantic sector have a close connection with the NAO variability, presenting as storms [2], floods [3], extreme rainfall [4], etc. The prediction skill of NAO is of great significance for climate prediction in North Hemisphere and has been a focus of the scientific subject.

The NAO index (NAOI), which is defined as the normalized sea level pressure difference between Iceland and the Azores, is adopted as an indicator to characterize the intensity of NAO events. In previous work for NAO prediction, the skills of proposed models are also reflected by the accuracy of mean NAOI. With the implementation of a 3D-Var assimilation system, the new version of the UK Met Office Global Seasonal forecast system (GloSea5) shows improved prediction for the NAO in the middle latitude [5]. Using the same high-resolution model, the latest generation seasonal prediction system called DePreSys3 enhanced the skill in one-year-ahead NAO prediction, and the skill source in the tropical Pacific region was also identified [6]. The impact on the NAO predictability of the Integrated Forecast System (IFS) caused by the regime dynamics of the North Atlantic eddy-driven has been explored, and the Markov model driven by seasonal persistence probabilities was constructed [7]. Although predicting NAO via numerical models is more mature, it still exists some obvious drawbacks. The errors implied in initial conditions along with those inherent to the model (for instance, parameter, precision, etc.), can lead to significant deviation on NAO prediction [8]. Besides, the physical mechanisms that are not generalized by the existing dynamical equations can also increase the uncertainty.

Owing to the limited capacity of most dynamical models in the seasonal prediction of the winter NAO, a new empirical model based on the multiple linear regression (MLR) techniques provided robust prediction for DJF (December, January, and February) mean NAOI, considering the impact of sea surface temperature (SST), sea ice concentration, and stratospheric circulation [9]. Selecting Pacific Ocean SSTs, sea ice in the Arctic, Atlantic SSTs, and tropical rainfall as predictors, a probabilistic prediction of the winter NAO has also been performed using linear regression [10]. However, the model did not work well on test sets and presented low reliability. The autoregressive integrated moving average model (ARIMA) combined with the extreme learning machine (ELM) [11], the statistical toy model based on Markov chain [12], and composite statistical models [13], like the polynomial-harmonic autoregressive model, threshold autoregressive model, and multivariate autoregressive model, have also been adopted to predict NAOI. Constrained by the simple mechanism embedded in these statistical models, the capacity of identifying the nonlinear feature is defective, causing a large deviation in prediction. As a complex air-sea nonlinear interaction, the NAO can hardly be described as the linear relationship between these physical variables. As a nonlinear fitting method, machine learning approaches can effectively avoid the above-mentioned defects by extracting features from data automatically and are widely adopted for predicting a variety of climate phenomena. Currently, the researches on NAO prediction using machine learning methods are still very few.

In addition to mid-term NAO predicted in previous works, our team also made an attempt on the short-term NAO forecasting using neural networks as well as mode decomposition methods, including ensemble empirical mode decomposition (EEMD) and discrete wavelet transform (DWT), which have been blended into models to improve the signal to noise ratio (SNR) [14, 15]. It is indicated that the accuracy on peak values, which normally represent extreme NAO events, has been notably enhanced. The forecasting result is compared with the two mature NAO forecasting products of CPC, which are Global Forecast System (GFS) and Ensemble Forecasts (ENSM), and our models present higher forecast reliability than these two products. The predictors adopted in these works only contain the factors directly related to the NAO (NAOI and SLP), and we aim to consider other variables with relevant physics meanings as the input for forecasting.

In related works for NAO prediction, vorticity, temperature, surface pressure, sea ice concentration and geopotential height have been selected as feature sources [16–18]. Among these predictors, SSTs have also found to be the crucial factor to trigger the NAO events [19]. For instance, the positive response of NAO can be forced by interference of climatological stationary wave, which is generated by Rossby wave from the SST warming [20]. In particular, the positive phase of NAO (NAO^+^) is associated with the positive SST anomaly located in the southeast of Newfoundland as well as the negative SST anomaly over the northeast of the North Atlantic [21]. The roles played by Pacific Ocean SST variability is found to be particularly beneficial to the summer NAO prediction, and the Pacific Ocean SSTs destructively interferes the climatological stationary wave by producing a Rossby wave, resulting in the positive NAO response [22]. Further, the causal relationships and interactions between ENSO and NAO are identified by correlation coefficient of NAOI and Niño index, demonstrating winter La Nina is more likely to drive the *NAO*^−^ events [23].

In this paper, prediction and forecasting of the NAO variability can be carried out based on the correlation between NAO and ENSO in two aspects. Firstly, the monthly NAOI variation is predicted by the RF-Var model, with selecting NAOI and Niño indices (including Niño3 index, Niño4 index, and Niño3.4 index) as inputs. On the other hand, the short-term NAO status is characterized by SLP and forecasted using the deep learning model AccNet. On the basis of the above work, in addition to physical variables that can define NAO directly, such as SLP and geopotential height (GH), the variables that have been proved to be closely related to the NAO variation, including zonal wind and meridional wind as well as SST are selected as predictors of the short-term NAO forecasting model. First of all, in order to investigate whether there exists a gain effect of SST in the tropical Pacific on NAO prediction and forecasting, this paper analyses the interaction details of the Niño3.4 index with NAOI in the decadal period using cross wavelet transform (XWT) and wavelet coherence methods. Wavelet transform is a traditional tool to analyze trends and periodicities with expanding time series into time-frequency space, and continuous wavelet transform (CWT) can be applied in the analysis of localized intermittent oscillations [24]. The causality between signals would be suggested by regions with large common power and consistent phase relationship [25]. Meanwhile, the rolling windowed time-lagged cross correlation (RWTLCC) method is adopted to determine the leader-follower relationship between ENSO and NAO. The analysis results show that ENSO has a driving effect on the evolution of NAO. For the mid-term NAOI variation prediction, the results show that the prediction accuracy of this method achieves 68%, which is better than other advanced classification methods, the regression model proposed by our team (DWT-LSTM and EEMD-ConvLSTM), and the prediction system (MATES1.0) based the on the numerical model. For the short-term SLP forecasting, the relevant physical variables, as listed above, including SLP, GH, winds, and SST, are fed into the multi-channel neural network model with trajectory gated recursive unit (TrajGRU) layers. Due to dynamic connections, the TrajGRU structure has shown high flexibility with ACC as the loss function to obtain the forecasting sequence of SLP. With forecasting 64 NAO^+^ events and 59 NAO^−^ events during the decade of 2010–2021, there is a certain degree of correlation between SST and different types of NAO events, and this correlation helps the model to learn the various characteristics of NAO, thus improving the forecasting skill of NAO.

The rest of the paper is structured as follows.  Section 2 introduces the related work on the correlation between ENSO and NAO and their combined effects. The dataset and regions we focus on are displayed in Section 3. The analysis tools and details of the RF-Var model and AccNet model are also presented in Section 3. Experiment settings including lead time settings and parameter settings are displayed in Section 4. The relevant analysis and results of NAOI prediction and SLP forecasting are discussed in Section 5. In the last section, we conclude with a summary and point out the future prospects.

## 2. Related Work

The ENSO phenomenon originates from coupled ocean-atmosphere circulation in the tropical Pacific Ocean and is a major cause of global interannual climate change. Because the correlation properties of ENSO and NAO provide potential seasonal predictive power for European climate, several previous results have been used to explore the influence of ENSO on NAO variability [26, 27]. The relationship between ENSO and NAO-related atmospheric circulation is complex, and one of the reasons for the complexity is the diversity of ENSO spatial structure, which is important for the seasonal prediction of NAO. In general, El Niño events in the Eastern Pacific (EP) and Central Pacific (CP) are often accompanied by the atmospheric response of *NAO*^−^. CP-type and EP-type ENSOs have different effects on NAO due to their unique regional climatic influences [28]. Among them, NAO^−^ events are more likely to be induced during El Niño, while NAO^+^ events are more likely to occur during La Niña [29]. These extratropical atmospheric responses are mainly attributed to nonlinear sea-air interactions in the tropical eastern Pacific. The influence of ENSO on NAO is highly seasonal, with the North Atlantic atmospheric anomalies in early winter (November-December) and late winter (January-March). However, the variations of ENSO in the SST anomaly modes are roughly opposite, and the diversity exhibited by ENSO in the SST anomaly modes also affects its correlation with NAO [30]. The atmospheric anomaly modes of NAO^−^ often coincide with El Niño events, and their common effect is a colder and drier late winter in Western Europe, while La Niña has roughly the opposite effect on NAO [31].

The combined effects of ENSO and NAO are confirmed to be more profound than the effects they produce individually [32]. For instance, the NAOI reached extreme negative values (<−4) during the winter of October 2009, when an El Niño event also occurred, leading to record snowfall in the mid-Atlantic region [33]. The typical El Niño event of 1982–1983 coincided with a NAO^+^ event, leading to heavy rainfall in southern China [34]. During 2009–2010, a drought occurred in southwest China, and the associated atmospheric anomalies were triggered by both NAO^−^ and El Niño [35]. However, the dynamic mechanisms of how ENSO-related tropical SST anomalies affect NAO variability have not been fully understood yet. Some studies have suggested that ENSO may cause SST anomalies in the North Atlantic Ocean, thus affecting the atmospheric circulation in the North Atlantic [36, 37]. Low-frequency atmospheric circulation anomalies over the eastern Pacific and North America regulate the meridional propagation of waves over the North Atlantic, which would trigger the generation of NAO events in different phases [31, 38]. During the period 1957–2007, a clear interdecadal feature of the correlation between ENSO and summer NAO emerged, and it is suggested that ENSO was significantly correlated with NAO after the mid-1970s [39]. It is also demonstrated that a poleward propagating Rossby wave enhanced by an SST anomaly of the Northwest Pacific associated with the ENSO development process was responsible for linking the ENSO signal to the NAO, causing the strongest winter NAO signal to coincide with the maturation of the ENSO [40]. Previous studies have indicated that negative SST anomalies in the northeast and southeast of the North Atlantic are correlated with NAO^+^, while lagged North Atlantic SST is significantly correlated with NAOI in the following winter [21, 41].

Doblas Reyes et al. adopted an ideal model to demonstrate that winter NAOI can be predicted on a one-month time scale [42], with pointing out the link between NAO and other external factors are crucial for the prediction of extreme climate events. Tian and Fan analyzed the time series of NAO using power spectra [43] and found that NAO exhibits spectral peaks in a 2 to 3 years cycle [44, 45]. ENSO and NAOI are chosen for the period 1948–2014 to determine the impact of different types of ENSO on climate change in the North Atlantic and concluded that the NAO^+^ is associated with winter CP-type La Niña, while the NAO^−^ is associated with winter EP-type La Niña [46]. Therefore, cross-validation tests and independent backward predictions of winter NAO were performed in the previous study using the SST of the previous spherical season and the year-to-year increment of the Eurasian snowpack as predictors [43]. The results show that the new prediction model exhibits better performance in reproducing the interdecadal variability of NAO.

## 3. Materials and Methods

For prediction and forecasting of the NAO, scholars generally focus on the occurrence and intensity of NAO events. And beyond that, the interannual scale variability of NAOI has also become a key point in related studies [47]. Therefore, NAO prediction and forecasting in this work will be carried out in two aspects. After exploring the correlation between ENSO and NAO, the first aspect is to select Niño indices and NAOI as predictors to predict the monthly NAOI fluctuation and variation trend using the RF-Var model; on the other hand, since the short-term NAOI can be manifested by SLP field in North Atlantic sector, physical variables associated with ENSO and NAO are fed into deep neural network named AccNet to forecast the SLP sequences.

### 3.1. Dataset and Region

NAOI and Niño3.4 index are selected to represent the trends of NAO and ENSO. Specifically, Niño3.4 index is the average value of SST anomaly (SSTA) in Niño3.4 region, which is the main observation region for El Niño or La Niña events, located at 170°W-120°W, 5°S-5°N, as shown in the red box line in Figure 1. The quantitative criterion for ENSO events is that if the 3-month moving average value of the Niño3.4 index is greater than or equal to 0.5°C (less than or equal to −0.5°C) for at least 5 consecutive months, it means that an El Niño (La Niña) event occur.

Since the indicators related to ENSO, including Niño1+2 index, Niño3 index, Niño3.4 index, Niño 4 index, the Oceanic Niño Index (ONI), and the Trans- Niño index (TNI), all use the month as the unit time scale, the monthly NAOI is selected to stay in step with the ENSO indicators. Thereinto, the Niño3.4 index is the most commonly used scientific measurement of ENSO, while Niño3 index and Niño4 index can be adopted to identify the type of ENSO [48].  Table 1 lists the status of the NAO corresponding to moderate and strong ENSO events at the same period [49], and the date in Table 1 represents peak periods during the ENSO event. According to the previous related work mentioned in section “Related Work,” the EP-type El Niño event occurred in the winter between 1982 and 1983 accompanies by a NAO^+^ event [34], and the CP-type El Niño event during the winter between 2009 and 2010 is also in connection with the NAO^−^ event [35]. Moreover, it is also proved that CP-type La Niña is closely associated with NAO^+^ and EP-type La Niña has close relation with NAO^−^ [46], which can be seen from Date 1973.12 and Date 2010.12. ENSO events mostly peak in winter, while the winter mode of NAO is also particularly prominent; the interaction between these two phenomena would be worth exploring. As the type and location of ENSO events make a difference to the impact of the NAO, the Niño3 index and Niño4 index are considered as predictors for NAOI variation prediction.

Thus, monthly average NAOI, Niño3.4 index, Niño3 index, and Niño4 index are selected for correlation analysis. The monthly average NAOI data is provided by the CPC website [50], and the monthly average Niño3.4 index, Niño3 index, and Niño4 index are provided by the NOAA website [51]. The time intervals of these two datasets are both from 1960-01 to 2021-10, and Figure 2 shows the indices in this time period. It can be seen that the frequency of NAO fluctuations is significantly higher than ENSO, which is due to the more rapid changes and more frequent vibrations of SLP compared to SST. According to historical data, a NAO^−^(NAO^+^) event may be likely to cause severe climate disasters when it is generated simultaneously with an El Niño event [35, 52, 53]. During the two decades 1990–2010, the changes of NAOI and Niño3.4/Niño3/Niño4 index seem to be a strong consistency. Whereas, before 1970, a more intuitive correlation feature cannot be captured.

As for the forecasting of grid-point data, some physical variables directly related to NAO, such as SLP and GH, are chosen as the predictors. The NAOI can be defined from the SLP anomaly (SLPA) projection on the NAO pattern. More specifically, the SLP field is subtracted from the climatological mean, then the SLP anomaly (SLPA) is projected on the NAO pattern (SLP_NAO_), and the NAOI is obtained:

(1) $$\begin{array}{c} \text{NAOI}=\frac{\langle {\text{SLPA,SLP}}_{\text{NAO}}\rangle }{\langle {\text{SLP}}_{\text{NAO}}{\text{,SLP}}_{\text{NAO}}\rangle }, \end{array}$$

where 〈·, ·〉 denotes the inner product operation of matrixes. Specifically, it is the sum of product for the corresponding elements of two matrixes. Similarly, the NAOI can be also calculated by the 300 hPa GH field:

(2) $$\begin{array}{c} \text{NAOI}=\frac{\langle {\text{GHA,GH}}_{\text{NAO}}\rangle }{\langle {\text{GH}}_{\text{NAO}}{\text{,GH}}_{\text{NAO}}\rangle }. \end{array}$$

From the research of NAO's optimal precursor in our previous work, the longitudinal wind (V-wind) and latitudinal wind (U-wind) are proved to contribute to the NAO evolution [54]. Therefore, SLP, GH, U-wind, and V-wind in the North Atlantic sector and SST in the tropical Pacific sector are selected as predictors. SLP, V-wind, U-wind and GH are provided by NCEP reanalysis data with a resolution of 2.5° × 2.5°, and the time interval is uniformly selected from 1981-09-01 to 2021-11-01 with daily time resolution, and the grid size of each frame is 25 × 53. SSTs are obtained from NOAA high-resolution SST daily value data with a resolution of 0.25° × 0.25° and are located in Niño3 (150°W-90°W, 5°S-5°N), Niño4 (160°E-150°W, 5°S-5°N), and Niño3.4 region, respectively. In order to fit with other variables, the SST data is firstly cropped and is zoomed out using quadratic-spline interpolation. Then the frame scale of SST is 25 × 53 as well.

### 3.2. Cross Wavelet and Wavelet Coherence

In this paper, the cross wavelet and wavelet coherence are adopted to explore the periodicity and lag phase of the causal relationship between ENSO and NAO. Weather or climate data generally consist of time series, and multiple traditional mathematical methods such as the Fourier transform, when studying the periodic properties of a series in the frequency domain, default to the underlying processes being stationary on the time scale. The wavelet transform, on the other hand, can extend the study of time series into the time-frequency space and can discover local periodicity. Among them, Continuous Wavelet Transform (CWT) is a common tool for analyzing local periodic oscillations in time series and is more suitable for feature extraction. According to the principle of Quepf Müller uncertainty, the temporal resolution of wavelets is inversely correlated with the frequency resolution, as in the case of Morlet mother wavelet:

(3) $$\begin{array}{c} \psi_{0}\left(\eta \right)=\pi^{-1/4}e^{i\omega_{0}\eta }e^{-1/2\eta^{2}}. \end{array}$$

where *η* is time and *ω* is frequency, and the idea of CWT is to use wavelets as filters and change the scale of the wavelets to act on the time series. A CWT with a uniform time step *δt* can be defined as the convolution of a time series *x*_*n*_ with a normalized wavelet as follows:

(4) $$\begin{array}{c} W_{n}^{X}\left(s\right)=\sqrt{\frac{\delta t}{s}}\sum_{n=1}^{N}x_{n\prime }\psi_{0}\left[\left(n\prime -n\right)\frac{\delta t}{s}\right]. \end{array}$$

The power synchronization relationship and phase relationship between two time series in the time-frequency space can expose the causal relationship between them. The cross wavelet transform *W*_*n*_^*XY*^(*s*), which consists of the continuous wavelet transforms *W*_*n*_^*X*^(*s*) and *W*_*n*_^*Y*^(*s*) of these two time series *x*_*n*_ and *y*_*n*_, can reflect their common power spectrum and relative phase, whose power is defined as |*W*^*XY*^|. The power of the cross-wavelet presents the region with high common power, and another measure is the coherence of the cross-wavelet transform, defined as follows:

(5) $$\begin{array}{c} R_{n}^{2}\left(s\right)=\frac{{\left|S\left(s^{-1}W_{n}^{XY}\left(s\right)\right)\right|}^{2}}{S\left(s^{-1}{\left|W_{n}^{X}\left(s\right)\right|}^{2}\right)\cdot S\left(s^{-1}{\left|W_{n}^{Y}\left(s\right)\right|}^{2}\right)}, \end{array}$$

where *S* is a smoothing operator and can be described as

(6) $$\begin{array}{c} S\left(W\right)=S_{\text{scale}}\left(S_{\text{time}}\left(W_{n}\left(s\right)\right)\right), \end{array}$$

where *S*_scale_ is the smoothing operator along the wavelet scale axis and *S*_time_ represents the smoothing operator on the time scale. For the Morlet wavelet, the smoothing operator designed by Torrence and Compo is as follows [55]:

(7) $$\begin{array}{c} S_{\text{time}}{\left(W\right)|}_{s}=\left(W_{n}\left(s\right)*c_{1}{}^{-t^{2}/2s^{2}}\right)|,\\ S_{\text{scale}}\left(W\right)|={\left(W_{n}\left(s\right)*c_{2}\Pi \left(0.6s\right)\right)|}_{n}, \end{array}$$

where *c*_1_ and *c*_2_ are constants, and Π is a rectangular function. XWT can be considered as a local correlation between two sets of CWTs. If there is a physical correlation between the two sequences, a consistent or slowly varying phase lag will be presented.

### 3.3. RF-Var Model

The RF-Var model is proposed to conduct the prediction of NAOI variations from the perspective of solving the classification problem based on the random forest approach. The procedure of the RF-Var model is displayed in Figure 3. First, subdatasets are constructed by taking put-back samples from the original dataset. Then the subdecision trees are constructed via these subdatasets, and each subdecision tree outputs its result. For the new data that needs to be classified by the RF-Var model, the result can be obtained by majority voting on the judgments of subdecision trees. From this, the predicted NAOI variation sequence is acquired.

Random forest is a supervised learning algorithm in which the forest is a collection of decision trees, and the main idea is to improve the overall accuracy by combining learning models. An important feature of random forests is the ability to measure the impact of each feature on the prediction and the interaction between different features, thus avoiding overfitting to some extent.

In this paper, the monthly variation prediction can be transformed into a binary classification problem by using 0 to indicate a decreasing NAOI and 1 to indicate an increasing NAOI. The original data needs to be processed first. Assuming a time window of *n* for the prediction, the current element of inputs including NAOI and Niño index, which is written as *X*_*c*_′, is processed by comparing *X*_*c*−*n*−1_ and *X*_*c*−*n*_ of the raw sequence. The output *Y* is determined by the NAOI variation. Specifically, *Y*_*c*_ is set to 1 when *X*_*c*−1_ < *X*_*c*_ in NAOI or *c*=0, otherwise *Y*_*c*_ is set to 0. Therefore, the predictions are accordingly rising (1) and falling (0) for the NAOI. In a piece of samples, features of NAOI and Niño index signals in the time window range are available for selection by the RF-Var model.

### 3.4. AccNet

The multivariate forecasting model AccNet is used to forecast the SLP grid-point data within several days, and the structure is schematically shown in Figure 4. The input to the model consists of SLP, SST, U-wind, V-wind, and GH. The multivariate variables are organized in the form of multi-channel time series and fed into the multivariate forecasting model AccNet, which consists of three parts: encoder-predictor-decoder, first extracting features in consecutive frames of the aforementioned time series using a CNN, then feeding into a trajectory gated recursive unit (Trajectory GRU, TrajGRU) [56].

As a structure for capturing spatio-temporal correlations, it has similar functions to the ConvLSTM, but the ConvLSTM uses a position invariant filter that cannot efficiently respond to continuous feature maps where the local structure changes, especially for variables such as SLP where there are frequent oscillations in the short term, and there are limitations to the effectiveness of the ConvLSTM. For general ConvRNNs, the state at position (*i*, *j*) at moment *t* is calculated as follows:

(8) $$\begin{array}{c} H_{t,:,i,j}^{\prime }=f\left(W_{hh}\text{concat}\left(\langle H_{t-1,:,p,q|\left(p,q\right)\in N_{i,j}^{h}}\rangle \right)\right)\\ =f\left(\sum_{l=1}^{\left|N_{i,j}^{h}\right|}W_{hh}^{l}H_{t-1,:,p_{l,i,j},q_{l,i,j}}\right), \end{array}$$

where *N*_*i*,*j*_^*h*^ denotes the ordered set of neighborhoods at position (*i*, *j*), (*p*_*l*,*i*,*j*_, *q*_*l*,*i*,*j*_) is the *l*^*th*^ neighborhood position at position (*i*, *j*), and *W*_*hh*_^*l*^ is the convolution weight between the states, represented in matrix form. The hyperparameters of the convolution are fixed, so the set of neighborhoods is also fixed. the advantage of TrajGRU is the adoption of a connection structure that changes dynamically with the position. the state at position (*i*, *j*) at moment *t* in TrajGRU is calculated as follows:

(9) $$\begin{array}{c} H_{t,:,i,j}^{\prime }=f\left(\sum_{l=1}^{L}W_{hh}^{l}H_{t-1,:,p_{l,i,j}\left(\theta \right),q_{l,i,j}\left(\theta \right)}\right), \end{array}$$

where *L* is the total number of connections and the *l*^*th*^ neighborhood position in the neighborhood set contains the parameter *θ*, noted as (*p*_(*l*, *i*, *j*)_(*θ*), *q*_(*l*, *i*, *j*)_(*θ*)). As a result, TrajGRU can generate the set of neighbors at the current moment based on the location information using the current input and previous states as follows:

(10) $$\begin{array}{c} U_{t},V_{t}=\gamma \left(X_{t},H_{t-1}\right),\\ Z_{t}=\sigma \left(W_{xz}*X_{t}+\sum_{l=1}^{L}W_{hz}^{l}*\text{warp}\left(H_{t-1},U_{t,l},V_{t,l}\right)\right),\\ R_{t}=\sigma \left(W_{xr}*X_{t}+\sum_{l=1}^{L}W_{hr}^{l}*\text{warp}\left(H_{t-1},U_{t,l},V_{t,l}\right)\right),\\ H_{t}^{\prime }=f\left(W_{xh}*X_{t}+R_{t}\circ \left(\sum_{l=1}^{L}W_{hh}^{l}*\text{warp}\left(H_{t-1},U_{t,l},V_{t,l}\right)\right)\right),\\ H_{t}=\left(1-Z_{t}\right)\circ H_{t}^{\prime }+Z_{t}\circ H_{t-1}. \end{array}$$

where *U*_*t*_ and *V*_*t*_ are the locally connected flow fields of the storage structure generation network *γ*, *W*_*hz*_^*l*^, *W*_*hr*_^*l*^, and *W*_*hh*_^*l*^ are the weights of the projected channels implemented by 1 × 1 convolution, and warp() selects the positions by a bilinear sampling kernel. Let *M*=warp(*L*, *U*, *V*), then we have

(11) $$\begin{array}{c} M_{c,i,j}=\sum_{m=1}^{H}\sum_{n=1}^{W}L_{c,m,n}\max\left(0,1-\left|i+V_{i,j}-m\right|\right)\max\left(0,1-\left|j+U_{i,j}-n\right|\right). \end{array}$$

Compared with the *K* × *K* ConvGRU, the number of parameters of TrajGRU is *O*(*L* × *C*_*h*_^2^) (*C*_*h*_ is the state channel size), which is smaller than the number of parameters of ConvGRU, *O*(*K* × *C*_*h*_^2^), enabling more efficient learning of these locally connected features.

As it can be seen in Figure 5, the convolution hyperparameter of normal ConvRNN is fixed, while TrajGRU has the different *N*_*i*,*j*_^*h*^ for different locations. Downsampling in the encoder is implemented using convolution, and upsampling in the decoder is implemented using deconvolution.

The loss function of the general model is defined by the MSE or L1 paradigm, and AccNet uses the Anomaly Correlation Coefficient (ACC), which is an indicator of geological forecasting skill, as a loss function to highlight the spatial correlation between forecast series. Since the closer the ACC is to 1, the higher the correlation between the output and the true value, the loss function of AccNet is expressed as follows:

(12) $$\begin{array}{c} L_{a}=1-\text{ACC}\\ =1-\frac{\sum_{i=1}^{n}\left(O\left(I_{i}\right)-C_{m}-C_{jc}\right)\left(O\prime \left(I_{i}\right)-C_{m}-C_{ac}\right)}{\sqrt{\sum_{i=1}^{n}\left(O\prime \left(I_{i}\right)-C_{m}-C_{jc}\right)\sum_{i=1}^{n}{\left(O\prime \left(I_{i}\right)-C_{m}-C_{ac}\right)}^{2}}}, \end{array}$$

where *C*_*m*_=∑_*i*=1_^*n*^*I*_*i*_/*n*, *C*_*jc*_=1/*n*∑_*i*=1_^*n*^(*O*(*I*_*i*_) − *C*_*m*_), *C*_*ac*_=1/*n*∑_*i*=1_^*n*^(*O*′(*I*_*i*_) − *C*_*m*_), where *I*_*i*_ denotes the input grid, *O*(*I*_*i*_) denotes the forecast frame, *O*′(*I*_*i*_) refers to the observation frame.

## 4. Experimental Settings

### 4.1. The Lead Time of NAOI Variation Prediction Using RF-Var

Before conducting the prediction, the lead time for the prediction needs to be determined. As the samples of NAOI and Niño indexes are monthly averaged data, this paper selects the best lead time for pre-experimentation over a 12-month period. The RF-Var model is compared to a variety of classification models including decision tree, multilayer perceptron (MLP), support vector classification (SVC), k-nearest neighbor (KNeighbor), and Adaboost, etc. The macro average accuracy within 12 months is shown in Figure 6. In the previous work on monthly scale variability, the variability of the atmosphere can be reflected by the precipitation [57]. It has been proved that the typical asymmetry precipitation is closely related to the half-year oscillation, and its periodogram shows higher spectral density at the period of 6 months and 12 months. It means that the dataset of monthly NAOI stands a good chance to have distinctive features at intervals of 6 months or 12 months. These features in the time domain can be identified and captured by the machine learning model, resulting in accuracy vibration around 6 months or 12 months. As for the lead time less than 6 months, the RF-Var model has relatively higher accuracy and achieves the best accuracy (68%) when lead time is 3 months, and the accuracy of other models are all over 50% at this time. Therefore, 3 months is selected as the lead time of the RF-Var model for NAOI variation prediction.

### 4.2. The Lead Time of SLP Forecasting Using AccNet

According to (1), the SLP forecasting lead time is related to the short-term period of NAO. Since the NAO can be viewed as the process with an e-folding period of about two weeks, the autocorrelation coefficient (ACF) and the partial autocorrelation coefficient (PACF) are used to determine the optimal lag coefficient over a 14-day period. ACF describes the correlation between a given time series and a lag series over consecutive time intervals, while PACF describes the correlation between two independent points, excluding the influence of other points in the series. To derive the effect of the data *X*_*n*−*k*_ on the output *X*_*n*_, the PACF result would exclude the effect caused by the points *X*_*n*−*k*+1_,…, *X*_*n*−1_. For the lag factor *k*, the ACF and PACF are expressed as follows:

(13) $$\begin{array}{c} {\text{ACF}}_{k}=\frac{\sum_{i=1}^{n-k}\left(X_{i}-\bar{X}\right)\left(X_{i+k}-\bar{X}\right)}{\sum_{i=1}^{n}{\left(X_{i}-\bar{X}\right)}^{2}\sum_{i=1}^{n}\left(X_{i}-\bar{X}\right)},\\ {\text{PACF}}_{k}=\frac{E\left[\left(X_{n}-\hat{E}X_{n}\right)\left(X_{n-k}-\hat{E}X_{n-k}\right)\right]}{E{\left[\left(X_{n-k}-\hat{E}X_{n-k}\right)\right]}^{2}},\\ \hat{E}X_{n}=E\left[X_{n}|X_{n-1},\ldots ,X_{n-k+1}\right],\\ \hat{E}X_{n-k}=E\left[X_{n-k}|X_{n-1}\ldots ,X_{n-k+1}\right]. \end{array}$$

The ACF and PACF for the original NAOI series over 14 days are shown in Figure 7, with the confidence interval set at 95%. The figure shows that as the lag factor *k* increases, the further apart the data are, the weaker the dependence reflected by the ACF and the inclusion of the combined effect of the prefix series. The PACF, on the other hand, reveals the correlation between two points separated by a distance *k*. The PACF of a smooth sequence gradually decays as *k* increases until it tends to 0, at which point the minimum lag factor *k* is obtained. In Figure 7, the PACF steadily tends to 0 when *k* is greater than 5. Therefore, the lead time of SLP forecasting is set to 5 days.

With lead time within three weeks, the root mean squared error (RMSE) and coefficient of determination (R-Squared, *R*^2^) for SLP forecasting in November 2020 is presented in Figure 8. The RMSE and *R*^2^ are defined as follows:

(14) $$\begin{array}{c} \text{RMSE}=\sqrt{\frac{1}{n}\sum_{i=1}^{n}{\left|X_{o}-X_{f}\right|}^{2}},\\ R^{2}=\frac{\sum_{i=1}^{n}{\left(X_{f}-\bar{X_{o}}\right)}^{2}}{\sum_{i=1}^{n}{\left(X_{o}-\bar{X_{o}}\right)}^{2}}, \end{array}$$

where *X*_*o*_ and *X*_*f*_ denote observation data and the forecasted value, respectively, and $\bar{X_{o}}$ is the mean value of the observation data. The lead time of 5 days achieves the lower error and higher correlation coefficient, and the forecasting skill decreases sharply when lead time is longer than 12. Forecasting with 14-day lead time is much lower than those of 10-day lead time and 7-day lead time, which is inconsistent with the previous conclusion of our work [58].

### 4.3. Parameter Settings

This subsection lists relevant parameters of the RF-Var model and AccNet model. As for the midterm and low-frequency NAOI variation prediction, there are four kinds of indexes and 742 samples. Since the sample scale is not very large, the parameters we mainly focus on are the number of decision trees and the ratio of features.

Figure 9 illustrates how the macro average accuracy changes with these two parameters as well as the execution time. From subfigure (a), it can be seen that the execution time increases with the tree number, and the accuracy increases to 68% when the number of trees is equal to or greater than 1600. In general, the model would be easy to under-fit if the tree number is too small, and the execution time would increase obviously if the tree number is too large. When the tree number is increased to a certain number, the model improvement would be small. In this figure, when the number of trees is larger than 1600, the accuracy is still sustained at 68%. Thus, the tree number is set to 1600 to weigh up the performance and efficiency. The other parameter is the feature ratio, which denotes the number of features to consider when looking for the best split. From this figure, the accuracy does not change with the feature ratio, and it may be because the number of features is not large. The feature ratio is set to 0.5 due to the less execution time.

The rest of the parameters in the RF-Var model are also listed in Table 2, including the maximum depth of the tree, the minimum number of samples for splitting node, the minimum number of samples in a leaf node, and the threshold for node splitting. Thereinto, the maximum depth of decision trees is dynamically determined. It means that the node would be expanded until all leaves contain less than *S*_min_ samples or all leaves are pure.

As for the AccNet model, each frame of fields for variables mentioned above is of size 25 × 53, and the lead time is 5 days according to Figure 7. The dataset is grouped into the form of (batch size, lead time, channel number, frame height, frame width). The channel number equals to the number of variables and is set to 5. To achieve higher flexibility and forecast the SLP sequences with arbitrary length, multi-step forecasting is conducted via the rolling mechanism. The 1 forecasted frame is obtained by feeding the input sequences with 5 frames and is stitched behind the previous input sequence with removing the first element. After *n* rounds, the forecasted outputs with *n* frames are acquired. The loss function is replaced by ACC instead of L1-loss or MSE, and Adam optimizer is selected for training and optimizing [59]. Referring to the previous work, the learning rate is set to 1 × 10^−4^, and the momentum is set to 0.5 [56]. To fit the computing resources, the training batch size is set to 16, and the number of workers in the data loader is set to 4 to accelerate loading batches. Since the height and width are both odd numbers and in low resolution, the encoder contains only 1 recurrent neural network layer, with a symmetrical structure in the decoder. The convolution layers and structures for downsampling and upsampling are inserted into the encoder and decoder to enlarge the receptive field. The number of filters is set to 64, and the leaky ReLU with a negative slope of 0.2 is chosen as the activation function [60]. The number of links in TrajGRU layer *L* is set to 13, which has been proved to outperform kernel with the size of 7 × 7 in ConvGRU. these settings are also consistent with the previous work [61]. The kernel size of convolution structure of *γ* from inputs to hidden layer is set to 3 × 3 in, while the kernel sizes of convolutional operations from inputs to flow from hidden layer to flow, and generating flow are all set to 5 × 5. The input is trained for 200 epochs, and the model with the best training loss is saved (10).

## 5. Results and Analysis

### 5.1. Lagged Correlation and Wavelet Coherence

In this paper, the RWTLCC method is adopted to explore the correlation with directionality between NAO and ENSO. The principle of this method is to take one signal as a reference and generate several sets of lagged series of another signal in multiple time windows and calculate the correlation between them. Since the Niño3.4 index shows more closely related to the Australian climate, and it has been used to classify ENSO conditions in National Climate Centre [62], the interaction between NAO and ENSO is represented by the correlation between NAOI and Niño3.4 index.

The time span of the data sample is as long as 60 years and the climate state varies greatly at different stages. Thus, this paper divides the NAOI and Niño3.4 indices into 6 groups with 10 years as a stage. The time-lagged correlations between the NAOI and Niño3.4 indices between 1960 and 1990 are shown in subplots Figures 10(a)–10(c), and similarly the correlations between them in 1990–2021 are shown in Figures 10(d)–10(f). The horizontal coordinate represents the relative offset of the signal on the time axis, and the vertical coordinate represents the number of equal-length time segments. As can be seen from the figure, each segment of the signal is divided into 15 intervals except for the last group, and each row reflects the intercorrelation effect of the relative offset from −4 to 3. In (a), for example, the high correlation (red) is concentrated at the position of offset <0, indicating that NAO is guiding its interaction with ENSO during 1960–1970s interactions, while in (b) this correlation fluctuates over time, starting at time step 9, when NAO's role switches from leading to following. The correlation displayed in the first half of (c), representing the period 1980 to 1990, is dominated by NAO. From time step 8 onward, the positively shifted lagged version of NAOI shows an extremely high correlation with the Niño3.4 index, especially for the lagged version with an offset of −4 and −3. The leading role of ENSO lasts from around 1980 to 1982 and around 1991 to 1993, and the high correlation also appears in around 1997 to 2000. Since then the leading role alternates frequently in (e), and the driving impact of ENSO is reflected around 2015 to 2017 in (f).

Compared to the correlation coefficient curves, RWTLCC demonstrates a more fine-grained variation in the intercorrelation relationship. This paper also uses wavelet coherence to measure the correlation of these two series in the time-frequency domain. As described previously, wavelet coherence is calculated using Morlet wavelets, while its statistical significance level is estimated by Monte Carlo simulation.  Figure 11 plots the wavelet coherence and the cone of influence for the NAOI and Niño3.4 index, which is the region of the wavelet spectrum where edge effects are more important. The cone shows regions with confidence levels greater than 95%, and the color differences in the plot indicate differences in power spectral density. As with the time window grouping in Figure 10, the wavelet coherence results are presented as 6 groups from 1960 to 2021. The arrows in the regions with coherence above 0.5 show the phase lag of the NAOI with respect to the Niño3.4 index. The time lag is in connection with the period. For instance, the arrow in a vertically upward direction indicates a quarter of the phase lag; the arrow with the direction of horizontal rightward indicates the same phase, while the horizontal-leftward arrow indicates the opposite phase.

As can be seen from Figure 11, the signal phase time variation between NAO and ENSO slightly differs in 0–2.6 years, and the region of stronger coherence is generally located within the 12 months component before 2000. While starting from 2002, the annual period component is more coherent and the coherence lasts for a longer time scale, indicating that the covariance between NAO and ENSO in the one-year component is enhanced. Since then, the coherence cycle gets longer, which becomes more than 12 months in (e) and more than 24 months in (f). In the (e) subplot, a mid-term correlation appears in the period from 2000 to 2010, showing an annual resonant cycle with a negative phase. It is consistent with the corresponding relatively higher correlation with a larger offset in the (e) subplot in Figure 10. While in subplot (f), a phase difference of about 90° indicates that the fluctuations of ENSO precede NAO by about 0.25 cycles.

From a seasonal perspective, the distribution of Figures 11(a), 11(b), 11(d), and 11(e) has a certain pattern, with the coherence largely concentrated in winter. In addition, especially in (a) and (e), with a negative phase coherence and ENSO activity preceding the NAO, which can also demonstrate that the NAO in winter during this period is influenced by the regulation of the ENSO, producing North Atlantic atmospheric anomalies and thus affecting snowfall in the European region [31].

From the above analysis, it is clear that there is a certain coherence between the changes of ENSO and NAO, and ENSO may be one of the triggers of NAO changes during the duration of the coherence, thus the SST characterizing the ENSO phenomenon can be used as a factor to predict NAO.

### 5.2. Prediction of NAO Variation Using RF-Var Model

In addition to the intensity of NAO as well as the peak and duration of NAOI, the trend of NAO is also an important indicator of interest to meteorologists [63]. In the previous section, the influence and driving effect of ENSO on NAO are initially verified. In this section, the NAOI and Niño indices are used as inputs to jointly predict changes of the NAO. Unlike the NAOI regression prediction in our previous work [14, 15], the RF-Var model is based on the random forest approach to achieve the variation prediction of NAO from the perspective of solving the classification problem.

In the pre-experiment, setting the lead time *n*=3 to obtain relatively more accurate results. With a lead time of 3 months, the RF-Var model is compared with various classifiers such as decision tree, MLP, SVC, KNeighbor, and AdaBoost. The accuracy and other metrics are shown in Table 3.

Here the precision rate represents the proportion of correct predictions where the prediction is a positive example, while the accuracy rate represents the proportion of correct predictions in the prediction results, and the recall rate denotes the proportion of positive examples in the sample that are predicted correctly. Assume that the precision rate is *P* and the recall rate is *R*. The formula for the F1 score is as follows:

(15) $$\begin{array}{c} F1=\frac{2*P*R}{P+R}. \end{array}$$

The macro average metrics in this table are calculated as an arithmetic average for each category *P* and *R*, while the weighted average is calculated using the proportion of samples from each category to the total as the weight. Since the test set size is set to 5% of the dataset, 37 samples are adopted for accuracy statistics. For the prediction using 37 samples, the RF-Var model is significantly better than the above-mentioned classifiers, with a macro average accuracy of approximately 68%. Details of the 37 samples predicted using the RF-Var model are shown in Figure 12. The RF-Var model achieved consecutive correct predictions for the range of sample numbers from 2 to 9, while the high-frequency oscillations of NAOI from 30 to 35 intervals, where several incorrect predictions are found. In general, the RF-Var model has strong predictive power for NAO variations.

The subject operating characteristic (ROC) curves for the 37 samples predicted using the above method are shown in Figure 13. The variation prediction of NAOI is a binary classification problem, and its prediction result contains four possibilities: true positive (TP), false positive (FP), true negative (TN), and false TP means the predicted outcome is up and the true situation is up; FP means the predicted outcome is up and the true situation is down; TN means the predicted outcome is down and the true situation is down; FP means the predicted outcome is down and the true situation is up. The *X*-axis of the ROC curve is the False Positive Rate (FPR), the *y*-axis is the True Positive Rate (TPR), which is calculated as

(16) $$\begin{array}{c} \text{TPR}=\frac{TP}{TP+FN},\\ \text{FPR}=\frac{FP}{FP+TN}. \end{array}$$

The dashed line between the points (0, 0) and (1, 1) represents the result of random classification, and the area under the curve (AUC) of the ROC curve is used to measure the superiority of the classifier. Obviously, the AUC equals 0.5 for random classification, and AUC is less than 0.5 for the curve under the dashed diagonal line. It indicates poorer effect and inferior to random classification, while the classifier with 0.5 < AUC < 1 has a certain utilization value, and the larger the AUC, the better the effect. From Figure 13, the classification effects are ranked as follows: RF-Var > decision tree = MLP = SVC = AdaBoost > KNeighbor > random classification (Actually, the curves for AdaBoost and KNeighbor do not coincide), and the RF-Var model outstrips other classifiers obviously. The AUCs of the above classifiers are calculated to be 0.6845 (RF-Var), 0.5962 (decision tree, MLP, SVC, and AdaBoost), and 0.5577 (KNeighbor), respectively.

For the four cases of binary classification, the confusion matrix of the above method is shown in Figure 14, where the *x*-axis represents the predicted result and the *y*-axis represents the actual situation. The 37 samples contain 13 rising data and 24 falling data. In comparison, all the classifiers outperformed the prediction of the rising case than the prediction of the falling case, and the RF-Var model has a higher correct rate than the other models in both types of states. As for the KNeighbor classifier, its prediction result in the rising category is slightly worse than that of the decision tree, MLP, SVC, and AdaBoost methods.

The NAOI variation prediction has also been conducted in different seasons, and the prediction results are displayed in Figure 15. The dataset is split into different seasons, including winter (December, January, February), spring (March, April, May), summer (June, July, August), and autumn (September, October, November), and separately predicted. With the same test size ratio of 0.05 and the best lead time of 5 months, the macro prediction accuracy achieves 91.67%, 53.33%, 56.67%, and 63.33%, respectively. Thereinto, the prediction skill in winter significantly surpasses those of other seasons. The accuracy of prediction in spring, summer, and autumn are roughly equal. The RF-Var model is fully satisfied with the requirements of NAOI variation prediction in winter, which has an even greater impact on global climate.

The prediction results have also been compared against several deep learning models proposed by our team [14, 15].  Figure 16 presents the prediction results of NAOI variation from 2019-01 to 2021–10. DWT-LSTM and EEMD-ConvLSTM are both regression models combined with multi-mode decomposition preprocessing and neural network layers, and their lead times are set as 3, which is consistent with the RF-Var model. Their outputs are converted into raise/drop sequences, and there are 34 prediction results. From Figure 16, there are 24, 20, and 18 correct predictions are obtained by the RF-Var model, the DWT-LSTM model, and the EEMD-ConvLSTM model, respectively, with the macro average accuracy of 70.18%, 58.82%, and 52.94%. Although DWT-LSTM and EEMD-ConvLSTM perform well on NAOI multi-step forecasting within a few days, they may provide less reliability in mid-term NAOI variation prediction than the RF-Var model can achieve.

For the same prediction period, RF-Var model is also compared with the numerical prediction provided by MATES1.0, which is prediction system focus on the mid-high latitude-polar atmospheric teleconnection, sea ice, and snow cover. From 2019-01 to 2021–10, MATES1.0 provides 27 prediction results, and their input fields derive from NCEP Seasonal Climate Forecasts (CFS) v2, Beijing Climate Centre Climate System Model (BCC_CSM), and ECMWF Seasonal Forecast system 4 (S4), which are shortened to CFS, BCC, and ES in Figure 17. With the lead time of 3 months, MATES1.0-CFS achieves 8 correct predictions, MATES1.0-BCC correctly predicts 11 times and MATES1.0-ES obtains 14 correct predictions, which correspond to the macro average accuracy of 29.24%, 40.00%, and 51.59%, respectively. The numerical model has slightly worse performance in predicting NAOI variation owing to the complexity of the mechanisms considered in the kinetic equations, and the predictive skills of the RF-Var model is more reliable than the NAOI regression model previously proposed by our team and the established prediction products based on numerical models.

### 5.3. Forecasting of SLP Using AccNet Model

In order to verify the forecasting effect of AccNet, this paper intends to forecast the SLP for two types of NAO event durations between 2010 and 2021. the distribution of NAO events is shown in Figure 18, red blocks indicate NAO^+^ events, blue blocks indicate NAO^−^ events, and the text of the color block shows the sequential days for the event. Here, a slightly more rigorous NAO judgment method is adopted: NAOI < −1.0 or NAOI > 1.0 maintains for 3 days or more, with a total of 123 sets of NAO events are obtained. Among them, 64 cases are NAO^+^ events and 59 cases are *NAO*^−^ events. The NAO^+^ events are mainly distributed in winter and spring while the NAO^−^ events are mainly distributed in summer and autumn.

Since there are numerous NAO events during the decade, this paper takes the NAO^+^ event from November 10, 2020, as an example to show the forecast results of AccNet and other deep neural network models during the event duration. As shown in Figure 19, the event lasts for 6 days, all of the models are able to form an SLP structure that is close to the observation value. However, the structural differences at the lower latitude and the boundary between the two pressure centers still can be found. Due to the more complex spatial distribution of the SLP in the later period and the extremely irregular structure of the pressure center, the performance of the three models in the latter frames of the forecast needs to be improved, especially for the variation of small-scale spatial features.

Figure 20 displays the difference between the forecast results of each model and the observed data. It can be found that the higher errors are concentrated in the last two days of forecasts. In addition, since the closer the difference is to 0, the lighter the color, it can be seen that the forecast error of AccNet is significantly smaller than that of ConvLSTM and CNN + RNN. Even in the first 4 frames where the effect is slightly better, there are overestimation and overfitting at locations of higher pressure in ConvLSTM. Although the structure of CNN + RNN in forecasting SLP in Figure 19 is similar to the observed values, the shortcomings for capturing temporal features results in a large error in pressure forecasting. It can be seen that the dynamic connection of the TrajGRU module inside AccNet has some advantages in spatial-temporal features learning.

In Table 4, the mean values of each evaluation indicator for forecasting the decade 2010 to 2021 by these three models mentioned above are counted. Thereinto, RMSE and the mean absolute error (MAE) are commonly used indicators, and the peak signal to noise ratio (PSNR), the structural similarity index measure (SSIM), and the Universal Quality Index (UQI) are indicators to measure the image quality. They also can be adopted to estimate the forecast bias of grid points. The definition of MAE and PSNR are shown as follows:

(17) $$\begin{array}{c} \text{MAE}=\frac{1}{n}\sum_{i=1}^{n}\left|X_{o}-X_{f}\right|,\\ \text{PSNR}=20\cdot log_{10}\left(\frac{{\text{MAX}}_{X_{o}}}{\sqrt{\text{MSE}}}\right),\\ \text{where MSE}=\frac{1}{mn}\sum_{i=0}^{m-1}\sum_{j=0}^{n-1}{\left[X_{o}\left(i,j\right)-X_{f}\left(i,j\right)\right]}^{2}, \end{array}$$

where *X*_*o*_ refers to the observation data, and *X*_*f*_ denotes the estimated value. MAX_*X*_*o*__ denotes the maximum of the observation data, and *m* × *n* is the size of each SLP pattern. A larger PSNR means better forecasting. SSIM can be calculated by:

(18) $$\begin{array}{c} \text{SSIM}={\left(\frac{2{\bar{X}}_{o}{\bar{X}}_{f}+C_{1}}{{\bar{X}}_{o}^{2}+{\bar{X}}_{f}^{2}+C_{1}}\right)}^{\alpha }{\left(\frac{2\sigma_{o}\sigma_{f}+C_{2}}{\sigma_{o}^{2}+\sigma_{f}^{2}+C_{2}}\right)}^{\beta }{\left(\frac{\sigma_{of}+C_{3}}{\sigma_{o}\sigma_{f}+C_{3}}\right)}^{\gamma }, \end{array}$$

where $\bar{X_{o}}$ and $\bar{X_{f}}$ are the mean value of the observation data and forecasting series, respectively. *σ*_*o*_ and *σ*_*f*_ denote the standard deviation of the ground truth and forecasting, respectively. *σ*_*of*_ denotes the covariance of the ground truth and forecasting. *α*, *β*, and *γ* refer to the weighting parameters of brightness, contrast, and structure, and their values are all set to 1. *C*_1_, *C*_2_, and *C*_3_ are constants. Assume that *C*_3_=0.5*C*_2_, SSIM can be simplified as

(19) $$\begin{array}{c} \text{SSIM}=\frac{\left(2\bar{X_{o}}\bar{X_{f}}+C_{1}\right)\left(2\sigma_{of}+C_{2}\right)}{\left({\bar{X}}_{o}^{2}+{\bar{X}}_{f}^{2}+C_{1}\right)\left(\sigma_{o}^{2}+\sigma_{f}^{2}+C_{2}\right)}. \end{array}$$

UQI is a metric that can measure the similarity between patterns of observation and forecasting, and it can be written as

(20) $$\begin{array}{c} \text{UQI}=\frac{4\sigma_{of}\left(\bar{X_{o}}+\bar{X_{f}}\right)}{\left({\bar{X}}_{o}^{2}+{\bar{X}}_{f}^{2}\right)\left(\sigma_{o}^{2}+\sigma_{f}^{2}\right)}. \end{array}$$

SSIM and UQI are both in the range of [−1, 1], and the closer to 1 SSIM and UQI are, the more reliable forecasting the model achieves. In all these metrics, AccNet achieves the best results among the three models, slightly better than ConvLSTM.

To examine the differences in the forecasting effectiveness of NAO event models for different phases, for AccNet and ConvLSTM with similar performance in Table 4, the RMSE frequency distributions of these two models for forecasting 64 *NAO*^+^ events and 59 NAO^−^ events are plotted in Figure 21. It can be seen that AccNet has a smaller range of RMSE distribution. In the NAO^+^ event cases, the RMSE frequency distribution of AccNet is mainly in the range of [2, 6], while that of ConvLSTM is in [3, 7]. For the NAO^−^ event, the high-frequency number range of AccNet is concentrated in [2, 4], while ConvLSTM is located in [3, 6]. For these two models, the forecasting effects of NAO^−^ events are slightly better than that of NAO^+^ events. Combined with the evaluation metrics for each spatio-temporal prediction model in Table 4, it shows that TrajGRU, a structural unit that aggregates states in the form of learning trajectories, is more flexible than the fixed connection structure of ConvLSTM and CNN + RNN in the highly diverse NAO event test set.

## 6. Discussion and Conclusions

NAO is the most dominant atmospheric circulation mode in the Northern Hemisphere during winter and has a profound influence on the weather in Eurasia and even the global climate. The causes of climate phenomena have become unstable and complex due to the dramatic climate changes and human activities in the last two decades. At the same time, physical mechanisms that have not yet been studied increase the difficulty of providing reliable prediction and forecasting. As an alternative to climate prediction and weather forecasting, deep learning methods show great potential.

In this paper, we demonstrate a midterm NAOI variation prediction model and short-term SLP prediction model that consider the correlation between ENSO and NAO. First, the correlation between ENSO and NAO is analyzed using monthly average NAOI and Niño3.4 historical series data, and the series from 1960 to 2021 are split into six groups at 10-year intervals, and the correlation details are explored using RWTLCC and wavelet coherence methods, respectively. The results show that the ENSO-guided NAO changes are dominated during 1980–1982 and 1991–1993. And the intensity and duration of the ENSO-NAO coherence are higher around 1997 to 2000. From 2015 to 2017, the evolution of NAO triggered by the fluctuation of ENSO showed a high correlation. The NAO variability near 1973.12 and 2010.12 has also been proved to be connected with ENSO events in the same period. The RF-Var method is used to transform the NAOI variation prediction into a binary classification problem, which could achieve 68% accuracy, outperforming other widely used classifier models, the regression NAOI prediction model, and models based on numerical models. For the grid-point SLP forecasting, in addition to SLP and GH, which are directly related to NAO, SST, which can characterize ENSO, and V-wind and U-wind, whose sensitivity was verified in our works for identifying the OPR of NAO, were chosen as inputs. The above variables are fed into AccNet for training, and AccNet is a deep neural network with a multi-channel and encoder-decoder structure. Moreover, AccNet uses ACC, which evaluates the spatial correlation of geological information, as its activation function, and shows excellent performance in forecasting NAO events during 2010–2021, effectively improving the forecasting skill of NAO^−^.

## Figures and Tables

**Figure 1:** Critical observation areas for El Niño or La Niña events.

**Figure 2:** NAOI, Niño3.4 index, Niño3 index, and Niño4 index series for the period 1960–2021.

**Figure 3:** Structure of RF-Var model for NAOI variation prediction.

**Figure 4:** Schematic diagram of the structure of the multivariate forecasting model AccNet.

**Figure 5:** Comparison between ConvLSTM and TrajGRU.

**Figure 6:** Macro average accuracy of multiple models at different lead times.

**Figure 7:** The ACF (a) and PACF (b) for daily NAOI sequence within 14 days with confidence bounds of 95%.

**Figure 8:** RMSE and *R*^2^ of SLP forecasting for lead time within three weeks.

**Figure 9:** The parameter of RF-Var model. (a) is the number of decision trees, and (b) is the ratio of features.

**Figure 10:** Lagged intercorrelation between NAOI and Niño3.4 index obtained by RWTLCC method from 1960 to 2021 (a) RWTLCC 1960–1970 (b) RWTLCC 1970–1980 (c) RWTLCC 1980–1990 (d) RWTLCC 1990–2000 (e) RWTLCC 2000–2010 (f) RWTLCC 2010–2021.

**Figure 11:** Wavelet coherence analysis of NAO and ENSO during 1960–2021. (a) XWT 1960–1970. (b) XWT 1970–1980. (c) XWT 1980–1990. (d) XWT 1990–2000. (e) XWT 2000–2010. (f) XWT 2010–2021.

**Figure 12:** Prediction results of 37 samples in Table 3 using the RF-Var model.

**Figure 13:** ROC curves corresponding to Table 3.

**Figure 14:** Confusion matrixes of prediction results for multiple classifiers (a) RF-Var (b) decision tree (c) MLp (d) SVC (e) KNeighbour (f) AdaBoost.

**Figure 15:** Confusion matrixes of prediction results for different seasons. (a) Winter (DJF). (b) Spring (MAM). (c) Summer (JJA). (d) Autumn (SON).

**Figure 16:** Prediction results of RF-Var model and deep learning models, such as DWT-LSTM and EEMD-ConvLSTM.

**Figure 17:** Prediction results of RF-Var model and MATES1.0.

**Figure 18:** Distribution of the two types of NAO events between 2010 and 2021.

**Figure 19:** Forecast results of multiple models for an NAO^−^ event from 2020-11-10 to 2020-11-15.

**Figure 20:** Difference between forecast results and observed data in Figure 20.

**Figure 21:** RMSE frequency distribution of AccNet and ConvLSTM forecasting of NAO events in Figure 18. (a) RMSE frequency of AccNet for NAO^+^. (b) RMSE frequency of ConvLSTMfor NAO^+^. (c) RMSE frequency of AccNet for NAO^−^. (d)RMSE frequency of ConvLSTMfor NAO^+^.

**Table 1:** Different ENSO events along with the NAO status.

Date	ENSO event	ENSO type	ENSO intensity	NAO phase	NAOI
1965.11	El Niño	EP	Moderate	NAO^−^	0.38
1971.01	La Niña	EP	Moderate	NAO^−^	−1.13
1972.11	El Niño	EP	Strong	NAO^+^	0.54
1973.12	La Niña	CP	Moderate	NAO^+^	0.32
1975.12	La Niña	CP	Moderate	—	0.00
1983.01	El Niño	EP	Very strong	NAO^+^	1.59
1987.08	El Niño	EP	Moderate	*NAO* ^−^	−0.83
1988.12	La Niña	EP	Strong	NAO^+^	0.61
1992.01	El Niño	EP	Moderate	NAO^−^	−0.13
1994.12	El Niño	CP	Moderate	NAO^+^	2.02
1997.11	El Niño	EP	Very strong	*NAO* ^−^	−0.90
2000.01	La Niña	EP	Moderate	NAO^+^	0.60
2002.11	El Niño	CP	Moderate	NAO^−^	−0.18
2008.01	La Niña	EP	Moderate	NAO^+^	0.89
2009.12	El Niño	CP	Moderate	NAO^−^	−1.93
2010.12	La Niña	EP	Moderate	NAO^−^	−1.85
2015.12	El Niño	EP	Very strong	NAO^+^	2.24
2020.11	La Niña	EP	Moderate	NAO^+^	2.54

**Table 2:** Parameters of RF-Var model.

Name	Description	Value
*d*_max_	The maximum depth of the tree	Dynamic
*S*_min_	The minimum number of samples required to split an internal node	2
*L*_min_	The minimum number of samples required to be at a leaf node	1
*t*_*s*_	The threshold for node splitting	0.0

**Table 3:** Prediction results of multiple classifiers.

Name		Precision	Recall	F1 score
RF-var	Raise (1)	0.60	0.75	0.67
	Drop (0)	0.76	0.62	0.68
	Macro avg	0.68	0.68	0.68
	Weighted avg	0.69	0.68	0.68

Decision tree	Raise (1)	0.43	0.69	0.53
	Drop (0)	0.75	0.50	0.60
	Macro avg	0.59	0.60	0.56
	Weighted avg	0.64	0.57	0.58

MLP	Raise (1)	0.43	0.69	0.53
	Drop (0)	0.75	0.50	0.60
	Macro avg	0.59	0.60	0.56
	Weighted avg	0.64	0.57	0.58

SVC	Raise (1)	0.43	0.69	0.53
	Drop (0)	0.75	0.50	0.60
	Macro avg	0.59	0.60	0.56
	Weighted avg	0.64	0.57	0.58

KNeighbor	Raise (1)	0.40	0.62	0.48
	Drop (0)	0.71	0.50	0.59
	Macro avg	0.55	0.56	0.54
	Weighted avg	0.60	0.54	0.55

AdaBoost	Raise (1)	0.43	0.69	0.53
	Drop (0)	0.75	0.50	0.60
	Macro avg	0.59	0.60	0.56
	Weighted avg	0.64	0.57	0.58

**Table 4:** Evaluation indicators of SLP forecasting using multiple models.

Model	RMSE	MAE	PSNR	SSIM	UQI
AccNet	5.13	3.96	11.93	0.59	0.90
ConvLSTM	5.78	4.60	11.18	0.56	0.84
CNN + RNN	10.67	8.85	6.99	0.39	0.80

## Data Availability

The monthly average NAOI data are provided by the CPC website (https://www.cpc.ncep.noaa.gov/products/precip/CWlink/pna/nao.shtml), and the monthly average Niño indices data are provided by the NOAA website (https://psl.noaa.gov/gcos_wgsp/Timeseries/). SLP, V-wind, U-wind, and GH are provided by NCEP reanalysis data with a resolution of 2.5°×2.5° and daily time resolution, and the grid size of each frame is 25×53. SSTs are obtained from NOAA high-resolution SST daily value data with a resolution of 0.25°×0.25° (for instance, and SLP is obtained by https://www.esrl.noaa.gov/psd/cgi-bin/db_search/DBSearch.pl?Variable=Sea+Level+Pressure&group=0&submit=Search).
